RETRACTED

# Clinicopathological Features and Prognostic-Related Risk Factors of Gastric Signet Ring Cell Carcinoma: A Meta-Analysis

**DOI:** 10.1155/2022/3473445

**Published:** 2022-08-05

**Authors:** Ying Guo, Qian Wang, Qing Tian, Changwen Bo, Na Li, Sujing Zhang, Peishun Li

**Affiliations:** ^1^Department of Oncology, The First Hospital of Hebei Medical University, Shijiazhuang, Hebei 050000, China; ^2^Thoracic Surgery Department, The First Hospital of Hebei Medical University, Shijiazhuang, Hebei 050000, China; ^3^Department of Oncology, Tengzhou Central People's Hospital, Tengzhou, Shandong 277500, China

## Abstract

**Background:**

Gastric signet ring cell carcinoma (SRCC) has shown a growth growing trend worldwide, but its clinicopathological features and prognostic-related risk factors have not been systematically studied. This systematic review was devoted to this.

**Method:**

PubMed, Embase, Cochrane Library, and Web of Science databases were retrieved, and retrospective cohort studies comparing clinicopathological features and related risk factors in SRCC patients were included.

**Results:**

In SRCC patient population, males were more than females (male, OR = 1.38, 95% CI: 1.20-1.60); N3 patients were more than N0-2 patients (N0-2, OR = 3.19, 95% CI: 1.98-5.15); M1 patients were more than M0 patients (M0, OR = 3.30, 95% CI: 1.88-5.80); patients with tumor > 5 cm were more than those with tumor (≤5 cm, OR = 7.36, 95% CI: 1.33-40.60). Patients with age < 60 years (age ≥ 60 years, OR = 1.03, 95% CI: 1.01-1.05), lymphatic vessel invasion (no, OR = 1.74, 95% CI: 1.03-2.45), T2 (T1, OR = 1.17, 95% CI: 1.07-1.28) and T4 (T1, OR = 2.55, 95% CI: 2.30-2.81) stages, and N1 (N0, OR = 1.73, 95% CI: 1.08-2.38), N2 (N0, OR = 2.24, 95% CI: 1.12-3.36), and N3 (N0, OR = 3.45, 95% CI: 1.58-5.32) stages had higher hazard ratio (HR).

**Conclusion:**

SRCC may occur frequently in male. Age, lymphatic vessel invasion, TN, and M stage may be risk factors for poor prognoses of SRCC patients.

## 1. Introduction

Gastric cancer is the second cause of cancer death worldwide, and patients in advanced stage have low survival and high recurrence rate [1–3]. More than 1 million people are newly diagnosed with gastric cancer worldwide each year; in 2018, about 783,000 people died of gastric cancer [4]. In the past few decades, a unique type of gastric cancer, gastric signet ring cell carcinoma (SRCC), has been increasingly developed in Asia, Europe, and the United States, representing 35-45% of new cases of adenocarcinoma [5, 6]. SRCC is a special histologic type among all gastric adenocarcinomas with myxoid changes [7]. SRCC is often diagnosed with lymph node metastasis, distant metastasis, or both [8]. Many patients relapse after radical surgical excision [9]. Currently, the treatment strategy of SRCC is based on the multidisciplinary collaborative concept, but some patients still develop drug resistance or have relapse and metastasis after treatment [10–12]. Overall, current treatments have limited benefit for the overall survival of patients with SRCC, with a median survival of 12 to 20 months [11, 13–15].

RETRACTED

SRCC faces a number of clinical challenges. Endoscopy and pathology are difficult to popularize in early screening, and most patients have progressed by the time they are diagnosed [6]. Preliminary trials of combination therapy for SRCC have produced conflicting results, and there is currently no treatment regimen for SRCC, with most chemotherapy regimens targeting common adenocarcinomas [16, 17]. In addition to these clinical challenges, there is growing recognition that the poor prognosis of SRCC may be closely related to particular biological behaviors [18, 19].

In recent years, important achievements have been made to help us understand the epidemiology, pathology, molecular mechanisms, treatment options, and strategies of SRCC [20]. Previous works revealed the clinicopathological features of SRCC and their effect on prognostic risk factors, but the conclusions are conflicting [21]. In some reports, SRCC is associated with better outcomes [5, 22–24], while another study found no difference in 5-year survival between patients with SRCC and other types of gastric cancer [25].

Therefore, we conducted a meta-analysis to compare the clinicopathological features of patients with SRCC and to analyze prognostic risk factors, hoping to provide reference for clinical diagnosis and treatment of SRCC.

## 2. Method

### 2.1. Literature Retrieval

The methodology of this study strictly followed the Preferred Reporting Items for Systematic Reviews and Meta-Analyses (PRISMA) [26]. Through searching databases of PubMed, Cochrane Library, Embase, and Web of Science, we collected all relevant literature from the inception of each database to October 2021. The keywords searched included “gastric signet ring cell carcinoma”, “clinicopathological features”, and “prognostic risk factors”. Since more keywords would narrow the scope of articles, the specific literature retrieval strategies were as follows: (gastric signet ring cell carcinoma [MeSH Terms]) OR (gastric signet ring cell carcinoma [Title/Abstract]). In the retrieval process, “signet ring cell carcinoma of stomach” was entered as the main retrieval keyword. Two investigators independently completed the literature retrieval, and disputes were solved by consultation with the third investigator.

RETRACTED

### 2.2. Literature Selection

Literature selection was completed by two investigators independently, and disputes were settled through consultation with a third investigator. The inclusion criteria were as follows: (1) SRCC was defined by the classification from World Health Organization (WHO) as the cancer with a more than 50% predominant signet ring cells (SRCs); (2) all patients were diagnosed with SRCC or had a history of SRCC; (3) at least one outcome of the following risk factors was reported, including sex, age, chemotherapy, and TNM stage; and (4) all included studies evaluated the clinicopathological features and prognostic significance of SRC histology in patients with gastric cancer and were designed as retrospective cohort studies. The exclusion criteria were listed as follows: (1) duplicate publications, case reports, reviews, conference abstracts, systematic reviews, case-control studies, meta-analyses, editorials, and letters; (2) studies without enough data to extract the results; (3) studies with only 1-3 references of randomized controlled trials, which was not enough to support the meta-analysis; and (4) studies failed to meet the classification from WHO.

### 2.3. Data Extraction and Quality Assessment

Data extracted from the literature included author information, year of publication, country, study design, sample size, and patient clinical features (sex, TNM stage, and tumor size), as well as data on comparisons in risk factors related to sex, age, chemotherapy, lymphatic vessel invasion, and TNM stage. Retrospective cohort studies were evaluated using the Newcastle-Ottawa Scale (NOS), which consists of 3 main components, including participant selection (4 stars), interstudy comparability (2 stars), and outcome assessment (3 stars). The total score was 9, and the literature with the score ≥ 6 was considered as good quality. Disagreements between the two investigators were resolved by the majority opinion after a third investigator evaluated all items involved.

### 2.4. Statistical Analysis

Stata version 16.0 was used for meta-analysis. When evaluating patients' clinical features and hazard ratio (HR), for dichotomous data, the odds ratio (OR) and 95% confidence interval (CI) were merged for analysis. *I*^2^ statistics was used to assess the statistical heterogeneity of the included studies. The fixed effect model was first selected for detection. If *p* > 0.1 or *I*^2^ < 50%, it was indicated that there was no heterogeneity, and the fixed effect model was used. If *p* < 0.1 or *I*^2^ > 50%, it was indicated that there was significant heterogeneity, and the random effect model should be used for detection.

RETRACTED

## 3. Results

### 3.1. Literature Retrieval and Study Selection

Based on the developed retrieval strategy, a total of 1,607 articles were retrieved, and 724 duplicated articles were excluded. By browsing titles and abstracts, 656 articles were discarded. The rest of 68 articles were read in full text, among which 48 articles reported irrelevant data, 8 articles did not have enough data to extract the results we wanted, and finally, 12 articles were included [18, 21, 27–36].  Figure 1 shows the literature screening process.

### 3.2. Study Features and Quality Assessment

A total of 12 articles involving 15,493 patients were included, all cohort studies.  Table 1 shows the characteristics and quality assessment results of all the included literature. The literature quality score of each study was 6 points or above, indicating the high quality of the literature.

### 3.3. Meta-Analysis of Clinicopathological Features

By investigating the relationship between clinicopathological features and SRCC, we revealed that SRCC mainly occurred in males (*I*^2^ = 85.0%, *p* < 0.001, OR: 1.38, 95% CI: 1.20–1.60, Figure 2(a)). In addition, for TNM stage (Figures 2(b)–2(d)), SRCC patients presented high statistical heterogeneity and mainly occurred in T4 stage (*I*^2^ = 99.0%, *p* < 0.001, OR: 1.45, 95% CI: 0.85-2.47), N3 stage (*I*^2^ = 98.6%, *p* < 0.001, OR: 3.19, 95% CI: 1.98-5.15), and M1 stage (*I*^2^ = 99.2%, *p* < 0.001, OR: 3.30, 95% CI: 1.88-5.80). Meanwhile, more SRCC patients had tumors > 5 cm (*I*^2^ = 99.5%, *p* < 0.001, OR: 7.36, 95% CI: 1.33-40.60, Figure 2(e)). In sum, in the SRCC patient population, there were more male patients and patients at N3 stage, M1 stage, and those with tumors > 5 cm.

### 3.4. Meta-Analysis of Risk Factors

Thereafter, we analyzed the risk factors affecting overall survival in patients with SRCC. SRCC was revealed to have high statistical heterogeneity in age (*I*^2^ = 67.5%, *p* = 0.009, Figure 3(a)), chemotherapy (*I*^2^ = 98.9%, *p* < 0.001, Figure 3(c)), lymphatic vessel invasion (*I*^2^ = 64.1%, *p* = 0.016, Figure 3(d)), and T3 (*I*^2^ = 77.9%, *p* = 0.004, Figure 3(f)), T4 (*I*^2^ = 79.8%, *p* = 0.002, Figure 3(g)), and N (*I*^2^ = 77.5%, *p* = 0.001, Figures 3(h)–3(j)) stages. Hence, we introduced a random effect model, and higher HR was found in age < 60 years (HR: 1.03, 95% CI: 1.01-1.05, Figure 3(a)), nonchemotherapy (HR: 0.93, 95% CI: 0.45-1.41, Figure 3(c)), and lymphatic vessel invasion (HR: 1.74, 95% CI: 1.03-2.45, Figure 3(d)). In addition, HR was higher in T3 stage (HR: 3.72, 95% CI: 0.03-7.40, Figure 3(f)) and T4 stage (HR: 2.55, 95% CI: 2.30-2.81, Figure 3(g)) in comparison with T1 stage. N1 stage (HR: 1.73, 95% CI: 1.08-2.38, Figure 3(h)), N2 stage (HR: 2.24, 95% CI: 1.12-3.36, Figure 3(i)), and N3 stage (HR: 3.45, 95% CI: 1.58-5.32, Figure 3(j)) had higher HRs over N0 stage. However, SRCC showed low statistical heterogeneity in sex (*I*^2^ = 36.6%, *p* = 0.137, Figure 3(b)), T2 stage (*I*^2^ = 38.0%, *p* = 0.184, Figure 3(e)), and M stage (*I*^2^ = 40.9%, *p* = 0.149, Figure 3(k)). Subsequently, HRs were found to be higher in T2 stage (HR: 1.17, 95% CI: 1.07-1.28) and M1 stage (HR: 3.13, 95% CI: 2.94-3.32) with fixed effect model analysis. Accordingly, we suggested that age, lymphatic vessel invasion, and TNM stage might be risk factors affecting the overall survival of SRCC patients.

RETRACTED

## 4. Discussion

The incidence of SRCC has been increasing obviously in recent years [5, 6]. There have been many studies on the clinicopathological features of SRCC and their influence on prognostic risk factors, but no consistent conclusions have been drawn [21]. Therefore, we conducted and meta-analysis on the clinicopathological features and prognostic risk factors of patients with SRCC.

Studies have found that SRCC is a poorly differentiated adenocarcinoma with high malignancy, unique clinical features, and low survival rate [18, 37, 38]. We studied on the clinical features of SRCC patients, and the results showed that there were more males than females in SRCC patients. In respect of N stage, the population of patients in N3 stage was larger than that in N0 to N2 stage. In terms of M stage, the population of patients in M1 stage was larger than that in M0 stage. In a single-center database retrospective analysis, TNM stage significantly influences the poor prognosis of primary SRCC [39]. Besides, higher stage was an independent risk prognostic factor for patients with SRCC [40, 41]. Consistently, by further analysis of risk factors affecting the overall survival in SRCC patients, we found that patients had higher HR at T2 and T4 stages over T0 stage; N1, N2, and N3 stages over N0 stage; and M1 stage over M0 stage. However, in other studies, the correlation between TNM stage and SRC prognosis remains controversial and may be related to gene mutation and the degree of invasion of SRC [42–44], which requires further analysis by combining multiple causes.

It is well known that SRCC patients with larger tumors have a poorer prognosis, which may be because larger tumors are coupled to greater depth of invasion, worse histological grade, higher risk of lymph node metastasis, and distant metastasis [21, 41, 45]. Our analysis showed that tumor size > 5 cm was more common in SRCC patients than in patients with tumors ≤ 5 cm. Larger tumors are strongly linked to lymph node metastasis and more common in patients with advanced gastric cancer and cause poorer prognoses [41, 46, 47]. Although tumor size was not evaluated as a risk factor for overall survival in patients with SRCC in this study, the results suggested that lymphatic vessel invasion caused a higher HR. The association of tumor size and lymph node metastasis is indicative of the association between larger tumors and poorer prognosis [41], but data collection remains necessary for further analysis. Therefore, less invasive gastric surgeries (such as endoscopic mucosal resection and endoscopic submucosal dissection) are more beneficial for patients with early SRC, and patients with advanced SRCC require more thorough surgical treatment [44]. Nevertheless, these conclusions still need to be treated with caution as the results of this analysis exhibited a large heterogeneity between studies.

RETRACTED

SRCC is frequently found in the mid and distal stomach and is highly prevalent in younger populations [48]. Efared et al. [49] found that in 183 patients with gastric cancer, the mean age of SRCC patients was lower than that of non-SRCC patients, which was consistent with the preliminary analysis of our systematic review. In addition, an increasing number of early-onset gastric cancers [50] have been detected in people younger than 45 years old, and patients with early-onset SRCC are more prone to lymphatic vessel invasion [51]. Early-onset patients have fewer surgical complications than late-onset patients because the previous group receives chemotherapy in a larger proportion, which is conducive to a better prognosis [51, 52]. Consistently, the results of this study are also indicative of a lower HR in SRCC patients receiving chemotherapy. However, the prognosis of patients with early-onset and late-onset diseases remains controversial and may be related to more factors, which calls for further analyses.

Other limitations also call for future discussion. First of all, the current evidence is not strong enough, all of which was based on retrospective investigation that might cause selection bias. Additionally, 10 of the 12 studies we included were from East Asian countries. Given the possible epidemiological and demographic differences between East and West, their data provided may not be a good representation for western populations. Hence, the clinical features and risk factors of SRCC patients from European and American countries may be different. Second, there was considerable heterogeneity among the included studies. More prospective randomized controlled trials are needed in the future to analyze and summarize the clinicopathological features and risk factors of SRCC accurately.

RETRACTED

Taken together, our conclusions manifested that SRCC is associated more with males, larger tumor size, and higher TNM stage. In addition, younger age, lymphatic vessel invasion, and higher TNM stage may be linked to the poor prognosis of SRCC patients.

## Figures and Tables

**Figure 1:** Flow chart of literature screening.

**Figure 2:** Forest plot was applied to assess different clinicopathological characteristics following SRCC and non-SRCC gastric cancer. (a) Sex, (b) T stage, (c) N stage, (d) M stage, and (e) tumor size.

**Figure 3:** Forest plot of the influence of (a) age, (b) sex, (c) chemotherapy, (d) lymphatic vessel invasion, (e–g) T stage, (h–j) N stage, and (k) M stage on SRCC.

**Table 1:** Basic information of the included literature.

Author	Year	Country	Study design	Sample size (*n*)	Sex		T stage		N stage		M stage		Tumor size		NOS
					Male	Female	T1–3	T4	N0–2	N3	M0	M1	≤5 cm	>5 cm	
Yang	2018	China	Cohort study	375	209	166	116	259	206	169	337	38	NA	NA	7
Zhou	2020	China	Cohort study	403	259	144	176	227	292	111	360	43	227	176	8
Guo	2020	USA	Cohort study	7149	3758	3391	5845	1304	6621	528	4794	2355	NA	NA	9
Shi	2019	USA	Cohort study	4638	2446	2192	2424	1188	3606	626	2647	1991	NA	NA	9
Chen	2018	China	Cohort study	347	181	166	315	32	335	12	341	6	NA	NA	8
Kunisaki	2004	Japan	Cohort study	54	28	26	NA	NA	51	3	NA	NA	NA	NA	9
KYUNG	2011	Korea	Cohort study	41	19	22	NA	NA	NA	NA	NA	NA	9	32	9
Kyoung-Joo	2013	Korea	Cohort study	205	149	56	NA	NA	NA	NA	NA	NA	NA	NA	6
Kao	2018	Taiwan	Cohort study	185	96	89	NA	NA	181	4	NA	NA	NA	NA	6
Li	2020	China	Cohort study	144	96	48	61	83	NA	NA	NA	NA	NA	NA	6
Tang	2020	China	Cohort study	266	182	84	137	129	181	85	NA	NA	187	79	8
Wang	2021	China	Cohort study	1686	879	807	1021	665	1125	561	1436	250	935	751	9

## Data Availability

The data used to support the findings of this study are available from the corresponding author upon request.
